# Mindfulness-Based Interventions for the Occurrence of Postpartum Depression in Elderly Primiparas

**DOI:** 10.1155/2022/4202676

**Published:** 2022-08-13

**Authors:** Rui Mei, Fan Peng, Jing Xiong, Chanyuan Liu, Xiu Liu, Fang Wang, Lu Lv

**Affiliations:** ^1^Department of Medical Administration, Wuhan Mental Health Center, Wuhan, China; ^2^Department of Rheumatology, Wuhan Traditional Chinese Medicine Hospital, Wuhan, China; ^3^Department of Acupuncture, Wuhan Traditional Chinese Medicine Hospital, Wuhan, China; ^4^Department of Pharmacy, Wuhan First Hospital, Wuhan, China; ^5^Department of Psychiatry, Wuhan Wuchang Hospital Nanhu District, Wuhan, China; ^6^Department of Obstetrics and Gynecology, Wuhan Wuchang Hospital, Wuhan, China; ^7^Psychosomatic Medical Ward, Wuhan Mental Health Center, Wuhan, China; ^8^General Affairs Section, Wuhan Mental Health Center, Wuhan, China

## Abstract

This study aimed to investigate the independent risk factors for the occurrence of postpartum depression (PPD) in elderly primiparas and the effect of mindfulness-based intervention (MBI) on improving the PPD. Two hundred cases of elderly primiparas who underwent delivery in our hospital from January 2016 to December 2019 were enrolled as study participants and divided into an occurrence group (*n* = 60) and a nonoccurrence group (*n* = 140) according to whether they developed PPD. The occurrence group was divided into a study group (*n* = 30) receiving MBI and a control group (*n* = 30) without any intervention. Independent risk factors influencing the occurrence of PPD were identified using univariate and multivariate logistic regression analyses. The effect of the intervention was also analyzed in the study group. Education level, marital status, household monthly income per person, sex of the newborn, milk volume, sleep quality, and relationship with in-laws were risk factors for the development of PPD. After the intervention, Five Facet Mindfulness Questionnaire scores were increased in the study group and were higher than in the control group (*P* < 0.05). The study group also exhibited higher 10-item Connor-Davidson Resilience Scale scores, lower Hamilton Depression Rating Scale and Schizophrenia Quality of Life Scale scores than the control group (*P* < 0.05). A variety of independent risk factors affected the occurrence of PPD in elderly primiparas, and MBI should be targeted clinically to reduce their negative emotions, increase psychological resilience, and improve their quality of life.

## 1. Introduction

The trend toward older parenthood looks set to continue since women have higher pursuits in their career. Influenced by China's late marriage and delayed childbearing policy, many women embraced motherhood at 30 or 40, and are being referred to as elderly primigravida. Childbirth has a significant impact on mothers with a shift in roles for family members [1]. However, this role shift can cause tremendous physical and psychological stress to the woman, and even postpartum depression (PPD). PPD is a type of psychological disorder that arises after childbirth in which women tend to experience depression, insomnia, emotional agitation, and even suicide and infanticide in severe cases [2]. According to statistics, the prevalence of PPD is about 10%–20%, which is twice as high as the general population suffering from depression [3, 4]. PPD not only affects women's physical and mental health, destroys couple and parent-child relationships, and even affects child development, bringing serious psychological and economic burdens to mothers and families and affecting their quality of life [5, 6].

Due to the high incidence of PPD, effective screening and diagnosis at an early stage and targeted interventions can reduce the risk of the disease [7]. However, the etiology of PPD is complex and the pathogenesis remains unclear. In 2015, Norhayati et al. analyzed 203 PPD studies published between 2005 and 2014, and most of the findings supported that psychological, physiological, social, and obstetric factors are all risk factors for PPD [8].

The aim of this study was to identify independent risk factors affecting the occurrence of PPD in elderly primigravida by comprehensively analyzing risk factors for PPD identified in existing studies, designing a questionnaire for the elderly primigravida admitted to our hospital, and performing univariate as well as logistic regression analysis on the collected data. The feasibility of this intervention method was analyzed through a MBI for women with PPD by evaluating their level of mindfulness, psychological resilience, and quality of life.

## 2. Materials and Methods

### 2.1. Baseline Data

By cluster sampling, 200 cases of elderly primigravida who underwent delivery in our hospital from January 2016 to December 2019 were included as participants and divided into an occurrence group (*n* = 60) and a nonoccurrence group (*n* = 140) according to whether they developed PPD.

The 60 cases of elderly primiparas suffering from PPD were divided into a study group (*n* = 30) and a control group (*n* = 30). The differences in baseline data between the two groups were not significant (*P* > 0.05) in terms of education level, marital status, household monthly income per person, and sleep quality.

Inclusion criteria: primiparas, age ≥35 years, full-term pregnancy, and normal delivery.

Exclusion criteria: the presence of psychiatric disorders, serious pregnancy complications, serious organic diseases, hormonal imbalances, and women on antidepressant medication or psychotherapy.

A personal profile was established for elderly primigravida, including information such as name, age, telephone number, and home address, and an informed consent form was signed by study subjects. The study was approved by the ethics committee of our hospital.

### 2.2. Methods

#### 2.2.1. Factors Influencing PPD in Elderly Primigravida

The possible factors associated with the occurrence of PPD were collected by exploring the literature, including age, literacy, mode of delivery, sex of the newborn, relationship with in-laws, relationship with husband, and household monthly income per person, and a questionnaire was developed.

One week after delivery, the investigators distributed the questionnaires to the mothers, using a uniform instructional language and explaining the precautions for filling them out. Mothers completed the questionnaires independently within 20 min. The investigators collected and checked the questionnaires, and a total of 200 valid questionnaires were collected.

#### 2.2.2. Effect of MBI on PPD

No intervention was given to mothers in the control group, and only regular telephone follow-up was conducted.

In the study group, the mothers were given MBI. A quiet room was set up as a training place, and a counseling team consisting of psychological medical staff was established. MBIs are offered twice in hospital and 5 times at home per week for a total of 8 weeks.

*(1) First stage*. The theoretical knowledge of MBI was introduced to make them understand the process of training. Introductory-level courses, such as mindful breathing and mindfulness meditation, looking up at the sky and feeling the breeze blowing, habit breaking intervention, etc. During the training process, the body and mind were kept relaxed and focused, and emotions stabilized. Mothers can gradually develop the ability to focus on mindfulness.

*(2) Second Stage*. Body scan meditation, mindful walking, sitting meditation, etc. are conducted. These trainings enable mothers to master meditation skills so that they can better handle negative emotions such as anxiety and depression in their daily lives and improve their self-control abilities. After the training, experiences were shared and discussed in group settings, and the changes in emotions and thoughts were observed.

*(3) Third stage*. The content of MBI was reviewed. Mothers were encouraged to integrate mindfulness into their daily lives and summarize the gains and feelings during the training.

### 2.3. Outcome Measurement

#### 2.3.1. Incidence of PPD

The Edinburgh Postnatal Depression Scale (EPDS) and the Hamilton Depression Rating Scale (HAMD) were used to determine whether participants developed PPD.

The EPDS contains 10 items of anxiety, fear, sadness, crying, insomnia, self-blame, self-harm, hobbies, mental status, and responsiveness, ranging from 0–30. Participants who scored ≥13 demonstrated the presence of depressive disorders, with higher scores associated with more severe depression [9, 10].

The HAMD contains 24 items, and participants scored ≥7 to demonstrate depressive tendencies and >17 to demonstrate depressive disorders [11].

#### 2.3.2. Univariate and Multivariate Logistic Regression Analysis of PPD

Based on the participants' answers, a univariate analysis was performed and the factor with *P* < 0.05 was associated with PPD.

The factors of interest from the univariate analysis were set as independent variables, assigned values, and then subjected to logistic regression analysis to determine the risk factors affecting PPD.

#### 2.3.3. Levels of Mindfulness in the Study and Control Groups after MBI

The Five Facet Mindfulness Questionnaire (FFMQ) was used to score the level of mindfulness in two groups before and after the intervention. The FFMQ scale contains 39 items analyzed on five dimensions: observation, description, aware actions, nonjudgment, and nonreactivity, with higher maternal scores indicating higher levels of mindfulness [12, 13].

#### 2.3.4. Levels of Psychological Resilience in the Study and Control Groups after MBI

The level of psychological resilience was assessed using the 10-item Connor-Davidson Resilience Scale (CD-RISC-10) before and after the intervention in two groups. The CD-RISC contains 10 items, and a higher score indicates a higher degree of psychological resilience [14, 15].

#### 2.3.5. Depressive Mood in the Study and Control Groups after MBI

The degree of depression in both groups was assessed before and after the intervention based on the HAMD. The HAMD contains 24 items. The higher score indicates the more severe depression.

#### 2.3.6. Quality of Life in the Study and Control Groups after MBI

The Schizophrenia Quality of Life Scale (SQLS), which is designed to assess the quality of life of patients with schizophrenia, was used to assess the quality of life in both groups. The SQLS contains 30 items distributed between three factors: psychosocial (15 items), motivation and vitality (7 items), and symptoms and side effects (8 items), with higher scores indicating poorer quality of life [16, 17].

### 2.4. Statistical Analysis

The collected data were approved and imported into Statistical Package for the Social Sciences (SPSS) 20.0 for statistical analysis (IBM, Armonk, NY, USA). Descriptive statistical analysis and *χ*^*2*^ test were used for univariate analysis, and *P* < 0.05 indicated a significant difference. Factors with significant differences by univariate analysis were included in a multifactorial logistic regression analysis to determine the independent risk factors for PPD.

## 3. Results

### 3.1. Incidence of PPD

Sixty-five of these participants scored ≥13. Of those 65 participants, 60 of them scored >17 on the HAMD. The prevalence of PPD was 30%, as evidenced by the presence of depressive disorders in 60 of the 200 case in the study.

### 3.2. Univariate Analysis of PPD

According to the occurrence of PPD, 200 participants were divided into two groups: nonoccurrence group (*n* = 140) and occurrence group (*n* = 60). According to the statistical results, there was no significant correlation between age, occupation, whether pregnancy was planned and mode of delivery with PPD in elderly primiparas (*P* > 0.05). Educational level, marital status, per capita household income status, sex of the newborn, milk volume, feeding pattern, maternal personality, quality of sleep, relationship with in-laws, and relationship with husband were correlated (*P* < 0.05) with the occurrence of PPD and were factors associated with the occurrence of depression (Table 1).

### 3.3. Multivariate Logistic Regression Analysis for PPD

The relevant factors identified in the univariate analysis were used as independent variables, and the occurrence of PPD was used as the dependent variable. The results showed that literacy, marital status, household monthly income per person, sex of newborn, milk volume, quality of sleep, and relationship with in-laws were factors influencing the occurrence of PPD (Table 2).

### 3.4. Comparison of Preintervention Indicators

Baseline data were not significantly different (*P* > 0.05) and were comparable between the study and control groups (Table 3).

### 3.5. Comparison of Mindfulness Levels after MBI

The total FFMQ scores in the control group (117.95 ± 10.77) and in the study group (114.48 ± 13.40) did not differ significantly (*P* > 0.05). After intervention, the FFMQ scores in the study group were higher compared to the preintervention ones, and the scores of each dimension were increased in the study group. However, nonreactivity scores were decreased in the control group (*P* < 0.05). The FFMQ scores differed significantly between the two groups (Figure 1).

### 3.6. Comparison of Psychological Resilience after MBI

CD-RISC-10 scores did not differ significantly (*P* > 0.05) between the two groups before the intervention, and they were higher in the study group and lower in the control group following the intervention, exhibiting significant differences in CD-RISC-10 scores (*P* < 0.05) (Figure 2).

### 3.7. Comparison of Depression after MBI

The difference in HAMD scores between the two groups was not significant (*P* > 0.05) before the intervention. After the intervention, HAMD scores decreased in the study group and increased in the control group compared to the preintervention (*P* < 0.05). HAMD scores differed significantly between the two groups after intervention (Figure 3).

### 3.8. Comparison of Quality of Life after MBI

The SQLS scores and total scores of the two groups were not significantly different before the intervention (*P* > 0.05) and were lower in the study group and higher in the control group than those before the intervention, showing a significant difference between the two groups (*P* < 0.05) (Figure 4).

## 4. Discussion

The prevalence of PPD within 6 weeks after delivery is as high as 66.5%, decreasing to less than 22% between 6 weeks and 1 year after childbirth [18]. Most adverse emotions such as depressed mood, irritability, loss of appetite, and insomnia that occur in the postpartum period will resolve on their own within 15 days after delivery. However, symptoms will worsen in 25% of primiparas who will develop depression or even postpartum psychosis [19, 20]. The common tool for screening PPD is EPDS, which enables early diagnosis and treatment of high-risk mothers to prevent the development of symptoms [21]. With the change in life concepts, late marriage and late childbirth have become the norm. As a special group, elderly primiparas are more prone to emotional stress and postpartum depression due to age-related factors. Therefore, it is particularly important to determine the inducing factors and find more effective intervention methods to reduce the proportion of postpartum depression among elderly primiparas.

With regard to the complex mechanisms of PPD, scholars have conducted many studies, and the results have shown that several factors such as social support, couple relationship, maternal personality, life stress, and stress of caring for the baby are risk factors for PPD [22, 23]. For mothers who develop PPD, psychological interventions are the preferred treatment modality [24] since medication will negatively affect the newborn during breastfeeding. MBI, as an option of psychological intervention, has been used in the treatment of depression. Studies have shown that MBIs can improve depression in the perinatal period [25].

In this study, 200 cases of elderly primiparas who underwent delivery in our hospital from January 2016 to December 2019 were enrolled as participants, and the risk factors affecting PPD were identified by multicategorical logistic stepwise regression analysis. Sixty women who developed PPD were grouped. The study group was given MBI, and the patients' mindfulness level and psychological resilience improved, and their quality of life also improved. Evidence has also shown that the degree of psychological resilience in depressed patients showed a positive correlation with quality of life, i.e., patients with higher psychological resilience had a better quality of life [26], which is consistent with the findings of this study.

In conclusion, literacy, marital status, monthly household income per person, sex of the newborn, milk volume, sleep quality, and relationship with in-laws were risk factors affecting the development of PPD.

The novelty of this study is that, for the first time, PPD in elderly primiparas was analyzed. The shortcomings are as follows: (1) due to the complex factors of postpartum depression and the small number of study samples, the identified factors affecting the development of PPD were limited. (2) Long-term follow-up results need to be verified.

## Figures and Tables

**Figure 1:** Mindfulness level scores before and after intervention. ^#^*P* < 0.05 for comparison within group before and after the intervention, ^*∗*^*P* < 0.05 for comparison between groups after the intervention.

**Figure 2:** Analysis of psychological resilience. ^#^*P* < 0.05 for comparison within group before and after the intervention, ^*∗*^*P* < 0.05 for comparison between groups after the intervention.

**Figure 3:** Comparative analysis of depression before and after intervention. ^#^*P* < 0.05 for comparison within group before and after the intervention, ^*∗*^*P* < 0.05 for comparison between groups after the intervention.

**Figure 4:** Comparative analysis of quality of life. ^#^*P* < 0.05 for comparison within group before and after the intervention, ^*∗*^*P* < 0.05 for comparison between groups after the intervention.

**Table 1:** Univariate analysis of postpartum depression (*n* (%)).

Factor	Occurrence group (*n* = 60)	Nonoccurrence group (*n* = 140)	*χ* ^2^	*P*

Age (years)				
35–39	37 (61.7)	91 (65.0)	0.203	0.653
>39	23 (38.3)	49 (35.0)		

Education level				
High school and below	11 (18.3)	45 (32.1)	9.513	0.009
Junior college	18 (30.0)	41 (29.3)		
Bachelor's degree and above	31 (51.7)	54 (38.6)		

Occupation				
Yes	42 (70.0)	105 (75.0)	0.539	0.463
No	18 (30.0)	35 (25.0)		

Marital status				
First marriage	27 (45.0)	95 (67.9)	9.224	0.002
Remarriage	33 (55.0)	45 (32.1)		

Household income per person				
<3000	28 (46.7)	25 (17.9)	22.070	0.000
3000–5000	22 (36.7)	53 (37.9)		
>5000	10 (16.6)	62 (44.2)		

Whether planning to get pregnant				
Yes	41 (68.3)	95 (67.9)	0.004	0.947
No	19 (31.7)	45 (32.1)		

Mode of delivery				
Vaginal delivery	38 (63.3)	96 (68.6)	0.521	0.470
C-section	22 (36.7)	44 (31.4)		

Sex of newborn				
Male	23 (38.3)	78 (55.7)	5.076	0.024
Female	37 (61.7)	62 (44.3)		

Milk volume				
High	11 (18.3)	27 (19.3)	13.105	0.001
Moderate	19 (31.7)	78 (55.7)		
Little or none	30 (50.0)	35 (25.0)		

Feeding pattern				
Hand-feeding	9 (15.0)	12 (8.6)	6.169	0.046
Mixed feeding	19 (31.7)	28 (20)		
Breastfeeding	32 (53.3)	100 (71.4)		

Maternal personality				
Introvert	12 (20.0)	25 (17.9)	6.332	0.042
Between introversion and extroversion	31 (51.7)	95 (67.8)		
Extrovert	17 (28.3)	20 (14.3)		

Quality of sleep				
Good	11 (18.3)	53 (37.9)	42.695	0.000
Fair	14 (23.3)	68 (48.6)		
Poor	35 (58.4)	19 (13.5)		

Relationship with in-laws				
Good	10 (16.7)	67 (47.8)	18.503	0.000
Fair	24 (40.0)	42 (30.0)		
Poor	26 (43.3)	31 (22.2)		

Relationship with husband				
Good	12 (20.0)	92 (65.8)	6.827	0.033
Fair	35 (58.3)	29 (20.7)		
Poor	13 (21.7)	19 (13.5)		

**Table 2:** Logistic regression analysis of postpartum depression.

Variables	*β*	SE	Wals	*P*	OR	95% CI for exp	
						Lower	Upper

Education level	0.137	0.841	7.643	0.011	1.147	1.022	4.417
Marital status	0.388	0.954	4.346	0.023	1.474	1.169	6.434
Household income per person (RMB)	1.568	0.670	5.486	0.019	4.799	1.292	17.830
Sex of newborn	0.267	0.915	4.132	0.019	1.306	1.089	4.693
Milk volume	1.783	0.548	10.580	0.001	5.945	2.031	17.423
Feeding pattern	0.872	0.475	3.369	0.066	2.393	0.943	6.073
Maternal personality	0.386	0.891	1.363	0.286	1.471	0.119	4.714
Quality of sleep	1.611	0.449	12.872	0.000	5.010	2.077	12.082
Relationship with in-laws	1.254	0.506	6.142	0.013	3.504	1.300	9.445
Relationship with husband	0.574	0.522	1.208	0.272	1.755	0.638	4.935

*Β*, standardized coefficient; SE, standard error; Wals, Wald statistic; *P*, probability level; OR, odd ratio, 95% CI for Exp, the OR value of the corresponding variable and its 95% confidence interval.

**Table 3:** Comparison of preintervention indicators (*n* (%)).

Factor	Control group (*n* = 30)	Study group (*n* = 30)	*χ* ^*2*^	*P*

Education level				
High school and below	6 (20.0)	5 (16.7)	0.603	0.740
Junior college	10 (33.3)	8 (26.7)		
Bachelor's degree and above	14 (46.7)	17 (56.7)		

Marital status				
First marriage	12 (40.0)	15 (50.0)	0.606	0.436
Remarriage	18 (60.0)	15 (50.0)		

Household income per person				
<3000	15 (50.0)	13 (43.3)	1.925	0.382
3000–5000	12 (40.0)	10 (33.3)		
>5000	3 (10.0)	7 (23.4)		

Sex of newborn				
Male	10 (33.3)	13 (43.3)	0.635	0.426
Female	20 (66.7)	17 (56.7)		
Milk volume				

Large	8 (26.7)	3 (10.0)	2.880	0.237
Moderate	8 (26.7)	11 (36.7)		
Little or none	14 (46.6)	16 (53.3)		

Quality of sleep				
Good	5 (16.7)	6 (20.0)	0.405	0.817
Fair	8 (26.7)	6 (20.0)		
Poor	17 (56.6)	18 (60.0)		

Relationship with in-laws				
Good	4 (13.4)	6 (20.0)	0.567	0.753
Fair	13 (43.3)	11 (36.7)		
Poor	13 (43.3)	13 (43.3)		

## Data Availability

The datasets used and analyzed during the current study are available from the corresponding author on reasonable request.
